RETRACTED

# Acupuncture elicits neuroprotective effect by inhibiting NAPDH oxidase-mediated reactive oxygen species production in cerebral ischaemia

**DOI:** 10.1038/srep17981

**Published:** 2015-12-10

**Authors:** Guang-Xia Shi, Xue-Rui Wang, Chao-Qun Yan, Tian He, Jing-Wen Yang, Xiang-Hong Zeng, Qian Xu, Wen Zhu, Si-Qi Du, Cun-Zhi Liu

**Affiliations:** 1 Acupuncture and Moxibustion Department, Beijing Hospital of Traditional Chinese Medicine affiliated to Capital Medical University, 23 Meishuguanhou Street, Dongcheng District, Beijing 100010, China

## Abstract

In the current study, we aimed to investigate whether NADPH oxidase, a major ROS-producing enzyme, was involved in the antioxidant effect of acupuncture on cognitive impairment after cerebral ischaemia. The cognitive function, infract size, neuron cell loss, level of superoxide anion and expression of NADPH oxidase subunit in hippocampus of two-vessel occlusion (2VO) rats were determined after 2-week acupuncture. Furthermore, the cognitive function and production of O_2_^−^ were determined in the presence and absence of NADPH oxidase agonist (TBCA) and antagonist (Apocynin). The effect of acupuncture on cognitive function after cerebral ischaemia in gp91phox-KO mice was evaluated by Morris water maze. Acupuncture reduced infarct size, attenuated overproduction of O_2_^−^, and reversed consequential cognitive impairment and neuron cell loss in 2VO rats. The elevations of gp91phox and p47phox after 2VO were significantly decreased after acupuncture treatment. However, no differences of gp91phox mRNA were found among any experimental groups. Furthermore, these beneficial effects were reversed by TBCA, whereas apocynin mimicked the effect of acupuncture by improving cognitive function and decreasing O_2_^−^ generation. Acupuncture failed to improve the memory impairment in gp91phox KO mice. Full function of the NADPH oxidase enzyme plays an important role in neuroprotective effects against cognitive impairment via inhibition of NAPDH oxidase-mediated oxidative stress.

Stroke, mainly ischaemic stroke, is one of the leading causes of death globally and a major cause of long-term disability^1^. Survivors are at particular risk of cognitive decline, with ≥30% prevalence 3 months after the stroke, and even minor stroke events have cognitive sequelae^2^,^3^. This serious disability imposes a large burden on patients, their families, the healthcare system, and society^4^.

The imbalance between the generation and clearance of ROS-induced oxidative stress is one of the major mechanisms involved in the pathologic processes of ischaemic stroke^5^,^6^. Overproduced ROS are believed to initiate neurodegenerative processes during cerebral ischaemia due to the oxidative damage in lipids, proteins, and nucleic acids^7^. Unfortunately, ROS-scavenging antioxidants have shown disappointing results in clinical trials despite promising results in pre-clinical experiments^8^. Targeting the source of ROS formation may be a novel therapeutic strategy for the inhibition of oxidative stress and ischemic stroke.

RETRACTED

Although multiple enzymes contribute to oxidative stress in various tissues or cells, recent studies have demonstrated that NADPH oxidase is a major ROS-producing enzyme in the brain under physiological conditions^9^. NADPH oxidase is composed of membrane (gp91phox and p22phox) and cytosolic (p40phox, p47phox, and p67phox) subunits coupled with the GTPase protein Rac1^10^. It recently emerged as a neuronal enzyme with a potential role in memory formation, because it was found to be localized to hippocampus^11^. Evidence suggests NADPH oxidase is activated in the hippocampus under chronic cerebral hypoperfusion, causing oxidative stress and consequential hippocampal neuronal death and cognitive impairment^12^. The up-regulated NADPH oxidase-meditated ROS overproduction exacerbates neuronal damage during ischaemic stroke^13^. Direct or indirect inhibition of NADPH oxidase function has been proved to be neuroprotective after ischaemic stroke^14^,^15^.

Studies have indicated that acupuncture is a new potential alternative to relieve poststroke cognitive impairment^16^. However, the mechanism of the neuroprotective effect of acupuncture remains unclear. Our previous study demonstrated that acupuncture has beneficial effects on spatial memory and antioxidant status through increasing the activity of ROS-scavenging antioxidants, superoxide dismutase (SOD) and glutathione peroxidase (GSH-Px), to clear ROS in the hippocampus of cerebral multi-infarction rats^17^. In the current study, we examined the hypothesis that the NADPH oxidase, a major ROS-producing enzyme, is involved in acupuncture-induced anti-oxidative effects on cognitive impairment after cerebral ischaemia.

## Materials and Methods

### Animals and Drugs

The experimental protocol was approved by the Ethics Committee for Animal Experimentation and performed according to the Guidelines for Animal Experimentation of Capital Medical University, Beijing, China. The experiments were carried out in accordance with the requirements of the Provisions and General Recommendations for Chinese Experimental Animals. In our study, we have made efforts to minimize the number of animals used and their suffering.

Adult male Wistar rats (8 weeks of age), purchased from Vital River Laboratory Animal Technology Co. Ltd (Beijing China), were cage-acclimated for 3 days prior to surgery in a temperature-controlled environment on a 12 h light/12 h dark cycle, with food and water adlibitum. All experimental rats weighed 300–320 g and were randomized into different groups.

RETRACTED

Mice lacking the gp91phox NADPH oxidase subunit (The Jackson Laboratory, Bar Harbor, ME) were included in further analysis the role of gp91phox in the anti-oxidative effect of acupuncture. The gp91phox knockout (KO) mice (weighing 20 ± 2 g; 12 weeks of age) were maintained in a C57BL/6 background (backcrossed more than 10 generations). Wild-type littermates (weighing 20 ± 2 g; 12 weeks of age) were used as controls in the experiment. Animals were genotyped by PCR assay using genomic DNA from mouse tails and the Extract-N-Amp Tissue PCR kit (Biocytogen) and then randomized into different groups.

The NADPH oxidase antagonist agent apocynin was administered through a tail vein 30 min before acupuncture treatment. On the basis of the data from a previous study^25^, the dosage for a body weight of 2.5 mg/kg was chosen. An NADPH oxidase agonist agent, tetrabromocinnamic acid (TBCA), was purchased from Tocris Bioscience (Bristol, Avon, UK) and injected at 1.4 mg/kg through a tail vein 30 min before acupuncture treatment.

### Experimental Protocol

#### Experiment I(for Rat)

To observe the therapeutic effect of acupuncture on cerebral ischaemia, we conducted the Morris water maze task to evaluate cognitive function, TTC to measure infarct volumes and Nissl staining to determine the neuron cell loss. The rats were randomly divided into normal (WKY), sham-operated (WKY + sham), two-vessel occlusion (2VO), acupuncture (2VO + Acu) and non-acupuncture (2VO + Non-Acu) groups (n = 10 for each group). In addition, the oxidative stress index was measured by the content of O_2_^−^ using DHE staining. Meanwhile, NADPH oxidase and its subunits were assessed by lucigenin-enhanced chemiluminescence assay, western blot and RT-PCR at the corresponding time point.

#### Experiment II(for Rat)

To determine whether an acupuncture-induced anti-oxidative effect was associated with NADPH oxidase, the rats were randomly assigned to 2VO + Acu, 2VO + Apocynin, 2VO + vehicle, 2VO + TBCA + Acu and 2VO + vehicle + Acu groups (n = 10 for each group). The vehicle group received 10 μl of 50% DMSO. 14 days after acupuncture treatment, the infarct sizes and O_2_^−^ production were measured by TTC and DHE staining in all the groups.

#### Experiment III(for mice)

To investigate the role of gp91phox in the anti-oxidative effect of acupuncture-mediated NADPH oxidase, the effect of acupuncture on spatial memory after cerebral ischaemia in gp91phox-KO mice was evaluated by the Morris water maze (MWM). Twenty male gp91phox KO mice and twenty wild-type (WT) C57/BL6 mice were divided into two groups: WT + vessel occlusion (VO), WT + VO + Acu, gp91phox KO + VO, and gp91phox KO + VO + Acu groups (n = 10 for each group).

RETRACTED

### Acupuncture treatment

After immobilization, the rats and mice were provided 75% alcohol disinfectant at the acupuncture sites and then acupunctured by the acupuncturist with needles (0.3 × 40 mm, Hwato, China). “Baihui” (DU20) and bilateral “Zusanli” (ST36) were selected for the acupuncture group. In the sham acupuncture group, bilateral stationary non-acupuncture points were selected as the control stimulating point. On the third day after the operation, acupuncture was administered once daily for 2 weeks (1 day rest after 6 days of treatment). The needles were perpendicularly inserted at acupuncture points and non-acupuncture points 5 mm deep for rats and 3 mm deep for mice. Detailed procedures are shown in Table 1. All acupuncturists were state-licensed and had at least 2 years of clinical experience. Normal, sham-operated, and 2VO groups were given the same time and same level catching-grasping stimulus as the acupuncture group. No animal died during the acupuncture treatment.

### Vessel occlusion operation

The rats were anaesthetized with 3.5% chloral hydrate. The bilateral common carotid arteries of rats or unilateral common carotid arteries of mice were exposed with a midline ventral incision, carefully separated from the vagal nerves, and permanently ligated with silk suture. The sham-operated animals were operated on in a manner similar to that for the operated rats except for the common carotid artery occlusion. Detailed procedures were undertaken as described previously^34^,^35^. During the operation, body temperature was maintained at 37.5 ± 0.5 °C.

### Behavioral testing with Morris water maze

In Experiment I and II, the Morris water maze consisted of a circular pool (160 cm in diameter, 40 cm in depth) whose interior was painted black. The water temperature was maintained at 23 ± 1 °C. The pool was divided into four quadrants, and a removable circular escape platform (10 cm in diameter) was introduced into one of the quadrants (target quadrant) at a depth of 2 cm below the surface of the water. Each rat was subjected to four training trials on each of five consecutive days. If a rat failed to find the submerged platform within 90 s, it was guided to the platform or placed onto it by the experimenter. The rat was allowed to spend 10 s on the escape platform and then relaxed for 5 min before the next trial began. On day 6, the probe trial was conducted by removing the platform for 90 s.

RETRACTED

In experiment III, the circular tank was 150 cm in diameter and 35 cm high for gp91phox-KO mice. A transparent platform 8 cm in diameter and 24 cm high was placed 1.0 cm below the surface of the water, which was kept at 20 ± 1 °C. Each mouse received four training trials on each of 3 consecutive days and one day for the probe trial. If a mouse failed to find the submerged platform within 60 s, an escape latency of 60 s was recorded. All data were collected digitally using a charge-coupled device camera placed directly over the pool and coupled with video tracking software (TopScanlite, USA).

### TTC staining

The fresh brain, after removal of the cerebellum, brainstem, and other areas was stored immediately at 20 °C for 20 min and then sliced into five uniform 2-mm sections. These sections were incubated in 2,3,5-triphenyltetrazolium chloride (TTC) at 37 °C for 30 min and then immersed in 4% paraformaldehyde for 30 min. Stained slices were photographed, and infarction size was calculated with the help of image analysis software. Brain infarct sizes (%) were presented by white infarct area/ whole slice area x100%.

### Nissl staining

After acupuncture treatment, the animals were anesthetized with intraperitoneal administration of sodium pentobarbital (40 mg/kg) and perfused via the left ventricle with normal saline followed by 4% paraformaldehyde in PBS, pH 7.4. Excised brain tissues were dehydrated and frozen in Optimal Cutting Temperature compound (OCT, Miles Inc., Elkhart, IN) and sectioned at 30 μm thickness, then stained with Nissl staining. Briefly, the sections were immersed in 0.2% Cresyl violet for 5 min and were covered with xylene-based mounting medium. Finally, Nissl-stained sections in the CA1 region of hippocampus were observed blindly by a second investigator using a light microscope (400× magnification; Olympus BX 41 microscope).

### Dihydrothedium (DHE) staining

DHE staining was used for measurement of superoxide production. Hippocampus tissue samples were homogenized and perfused with 10 ml saline solution. These sections were incubated at 37 °C and protected from light for 30 min after adding the DHE reagent (GENMED). The fluorescence intensity was measured with an excitation wavelength of 540 nm and an emission wavelength of 590 nm.

### NADPH oxidase activity assay

Lucigenin-enhanced chemiluminescence was performed to measure the enzymatic activity. Hippocampus tissues were homogenized and then centrifuged at 4 °C for 20 min. After dark adaptation, the chemiluminescence value was recorded at 30-s intervals over 10 min using a luminometer and reported as relative light units per minute normalized to protein concentration. Protein concentration in the supernatants was determined using a Micro BCA protein assay (Thermo Scientific, USA).

RETRACTED

### Western blot analysis

We observed changes in the protein expression of NADPH oxidase subunits after acupuncture via western blot analysis. The hippocampus samples were homogenized and centrifuged for 10 min at 4 °C. Protein concentration in the supernatants was determined using a Micro BCA protein assay (Thermo Scientific). The protein samples were resolved by SDS-PAGE gels (Applygen) and transferred to PVDF membranes. After being blocked with 5% skim milk at room temperature for 1 h and washed four times for 5 min each time in TBST, blots were subsequently incubated with anti-gp91phox (1:5000; Epitomics), anti-p47phox (1:200; Santa Cruz Biotechnology), or anti-p67phox (1:100; Santa Cruz Biotechnology) overnight at 4 °C. After being washed, the membranes were further incubated with a secondary antibody (1:10000; KBL) for 60 min. The average intensity values of protein bands were scanned and analysed by an infrared imaging system (Odyssey). β-actin or GAPDH was used as the control for gel loading and protein transfer.

### Real-time reverse transcription-polymerase chain reaction (RT-PCR)

We further investigated whether the effect of acupuncture is related to the mRNA expression of NADPH oxidase in rats with cerebral ischaemia. Total RNA was extracted from the hippocampus using Trizol Reagent (Invitrogen) according to the manufacturer’s instructions. Primers used in this study were as follows: gp91phox, 5′-CAG GGG TTC CAG TGC GTG TTG CTC AAC CAG A-3′ (forward primer), 5′-GGT ACA GGA ACA TGG GAC CCA CTA TCC ATT TCC AAG -3′ (reverse primer) and GAPDH, 5′-TCC ATG ACA ACT TTG GCA TC-3′ (forward primer), 5′-CAT GTC AGA TCC ACC ACG GA-3′ (reverse primer). The mRNA levels were normalized to the housekeeping gene GAPDH, and quantification was performed using the efficiency-corrected ΔΔCt method.

### Statistical Analysis

Data analysis was performed with SPSS software version 16.0. All values are presented as the mean ± SEM. Parameters for spatial memory, including escape latency, swimming distance, and swimming speed, were analysed by two-way repeated-measures ANOVA followed by a post hoc least significant difference multiple comparison test. One-way ANOVA was conducted to compare the results of TTC staining, DHE staining, lucigenin-enhanced chemiluminescence assay, western blot analysis, PCR and the probe trial of MWM followed by a post hoc least significant difference multiple comparison test. A P value less than 0.05 was considered statistically significant.

## Results

### Acupuncture ameliorated ischaemia-induced cerebral impairment

Time latency, swimming distance, swimming speed and the percentage of time spent in the target quadrant were measured in the water maze task. Acupuncture treatment significantly decreased the total time spent in the hidden platform area during the (*p* < *0.0001*, Fig. 1a) and total distance travelled to reach the platform (*p* = *0.009*, Fig. 1b), suggesting that acupuncture could ameliorate the spatial memory impairment induced by cerebral ischaemia. A significant difference was observed between the 2VO + Acu and 2VO + Non-Acu groups (*p* = *0.043 and p* *=* *0.041*, Fig. 1a,b). One-way ANOVA did not reveal any significant differences among the four groups for swimming speed (*p* = *0.764*, Fig. 1c), indicating that cerebral ischaemia-induced cognitive impairment did not result from motor function impairment.

RETRACTED

In the probe trial, % time travelled in the target quadrant was significantly increased in rats with cerebral ischaemia receiving acupuncture treatment (*p* = *0.019*, Fig. 1d), and significant differences were found between the 2VO + Acu and 2VO + Non-Acu groups (*p* = *0.015*, Fig. 1d).

### Acupuncture attenuated cerebral ischaemic injury

Infarct sizes were assessed by TTC staining. Compared with the 2VO group, acupuncture treatment significantly reduced the infarct volume (*p* = *0.008*, Fig. 2 a,b). Significant differences were found between the 2VO + Acu and 2VO + Non-Acu groups (*p* = *0.009*, Fig. 2b).

Neuron cell loss was assessed by Nissl staining. Compared with the 2VO group, acupuncture treatment reduced neuronal cell loss (*p* < *0.0001,* Fig. 2e,f). Differences were observed between the 2VO + Acu and 2VO + Non-Acu groups (*p* < *0.0001,* Fig. 2e,f).

### Acupuncture suppressed NADPH oxidase-derived O_2_^**−**^ generation

Whereas overproduction of ROS leading to oxidative stress is one of the major mechanisms involved in the pathologic processes of ischaemic stroke, we aimed to investigate whether the beneficial effects of acupuncture were through the regulation of O_2_^−^ generation. Using DHE staining, we found that O_2_^−^ production in the hippocampus was significantly increased in the 2VO group in comparison with the WKY groups (*p* = *0.016*, Fig. 2c). This over-generated O_2_^−^ was markedly suppressed by the 2-week acupuncture treatment (*p* = *0.021* Fig. 2c). A significant difference was observed between the 2VO + Acu and 2VO + Non-Acu groups (*p* = *0.032*, Fig. 2c). These results suggested that acupuncture could attenuate cerebral ischaemic injury through meditating O_2_^−^ generation.

As recent studies have demonstrated that NADPH oxidase is a major O_2_^−^-producing enzyme in cerebral ischaemia, we aimed to investigate whether the suppression of O_2_^−^ generation in the acupuncture treatment group was associated with NADPH oxidase activation. Our results found that the increased NADPH oxidase activity induced by cerebral ischaemia was significantly suppressed by both acupuncture treatment at acupuncture points and non-acupuncture points (*p* = *0.044 and p* = *0.041*, Fig. 2d). These results demonstrated that acupuncture could suppress NADPH oxidase-derived O_2_^−^ generation.

RETRACTED

### Acupuncture decreased the expression of NADPH oxidase subunits

Given that NADPH oxidases play a role in acupuncture treatment, it is of interest to better define this target, that is, which catalytic subunit, gp91phox, gp47phox, or gp67phox, is relevant. To investigate this, we applied western blot to further analyse NADPH subunit expression in all groups. Our results showed that the protein levels of NADPH subunits p47phox, p67phox, and gp91phox were significantly increased in the hippocampus of rats after the 2VO operation (*p* = *0.021, p* = *0.033 and p* = *0.022*, Fig. 3a–c). Acupuncture treatment significantly attenuated the elevations of gp91phox and p47phox but not p67phox (*p* = *0.028, p* = *0.009*, and *p* = *0.082*, respectively, Fig. 3a–c). The protein level of gP91phox showed significant difference between acupuncture and non-acupuncture groups (*p* = *0.011,* Fig. 3c). RT-PCR was performed to analyse whether acupuncture regulated the NADPH oxidase activation through gp91phox mRNA in the hippocampus. In contrast with protein expression, no differences in gp91phox mRNA were found among all experimental groups (*p* = *0.075*, Fig. 3d). We concluded that the beneficial effects of acupuncture may result from the suppressed expression of NADPH oxidase subunits.

### The NADPH antagonist mimicked the antioxidant potential of acupuncture and The NADPH oxidase agonists reversed the beneficial effect of acupuncture

Given that the antioxidant effects of acupuncture were mediated by NADPH oxidase, we reasoned that an NADPH antagonist may mimic acupuncture on improving the cognitive competence. The time latancy, swimming speed and % time in target quadrant were measured in the water maze task. As shown in Fig. 4a–c, the improvement of spatial memory and learning abilities in 2VO + Apocynin and 2VO + vehicle + Acu groups were similar to 2VO + Acu group. However, the 2VO + TBCA + Acu and 2VO + vehicle groups failed to improve the spatial memory and learning abilities in comparison with 2VO + Acu group.

Moreover, apocynin administration reversed the elevation of O_2_^−^ and reduced infarct volume compared with the 2VO + vehicle group (*p* = *0.020 and p* = *0.028*, Fig. 4d–f), which was similar to the results of the acupuncture group (*p* = *0.799 and p* = *0.442*, Fig. 4d–f). NADPH oxidase agonist TBCA administration abolished the beneficial effect of acupuncture by significantly increasing infarct sizes and O_2_^−^ production in the 2VO + TBCA + Acu group compared with the 2VO + Acu group (*p* < *0.0001 and p* < *0.0001*, Fig. 4d–f). Together, these results suggest that NADPH antagonists mimic the antioxidant potential of acupuncture and that NADPH oxidase agonists reverse the beneficial effects of acupuncture.

RETRACTED

### Acupuncture required the full function of the NADPH oxidase enzyme to protect against cognitive impairment

The results of the behavioural testing are summarized in Fig. 5. No differences in swimming speed were observed among the four groups (*p* = *0.087,* Fig. 5c). Compared with the WT-VO group, the 2-week acupuncture treatment not only decreased the rise induced by cerebral ischaemia in escape latencies and swimming distances (*p* = *0.027 and p* = *0.011,* Fig. 5a,b) but also raised the percentage of time spent in the target quadrant (*p* = *0.040*, Fig. 5d), indicating that memory impairment was reversed by acupuncture. We further detected that gp91phox KO mice after cerebral ischaemia showed more impairment in spatial memory than the WT-VO group, which was evidenced by longer latencies (*p* = *0.019*, Fig. 5a), swimming distances (*p* = *0.015*, Fig. 5b) and the low percentage of time spent in the target quadrant (*p* = *0.026*, Fig. 5d) compared with the WT-VO group. Nevertheless, acupuncture treatment failed to improve the memory impairment in gp91phox KO mice (*p* = *0.069*, Fig. 5a–d), indicating that acupuncture does require full function of NADPH oxidase enzymes to protect against spatial memory deficits.

## Discussion

The present study demonstrated that acupuncture markedly attenuated oxidative stress in the hippocampus of rats after two-vessel occlusion as shown by the reduction of superoxide anion. Meanwhile, acupuncture significantly ameliorated the memory impairment induced by cerebral ischaemia, as shown by the decrease in time and distance to reach the hidden platform in the water maze task. The neuron cell loss and infract size were significantly reversed by acupuncture treatment. Thus, the protective effects of acupuncture against cerebral ischaemia injury appear to be at least in part associated with the significant decrease in cerebral oxidative stress.

We investigated whether acupuncture inhibited reactive oxygen species production via NADPH oxidase, the major O_2_^−^-producing enzyme. Our results indicated that acupuncture treatment could suppress NADPH oxidase activity induced by cerebral ischaemia. Acupuncture at non-acupuncture points had a similar effect on NOX activity to that performed at acupuncture points. Indeed, whether there is a difference between the acupuncture group and non-acupuncture group varies and arouses controversy. Some recent large acupuncture trials indicated that acupuncture and sham procedures at non-acupuncture points were not different in efficacy^18^,^19^, whereas more other studies have produced opposite conclusions^20^,^21^. However, there was still significant improvement in cognitive impairment, NOX activity, neuron cell loss and infract size in the 2VO + acu group compared with the 2VO group, which indicated that acupuncture has a neuroprotective effect on cerebral ischaemic injury.

RETRACTED

Moreover, we found that acupuncture downregulated the overexpression of the membrane-bound subunit gp91phox and cytosolic subunit p47phox without significantly affecting the level of mRNA expression. Therefore, the attenuation of cerebral oxidative stress induced by acupuncture might be partially attributed to NADPH oxidase inactivation. The NADPH oxidase antagonist agent apocynin mimicked the effect of acupuncture on ameliorating the cerebral impairment, decreasing infarct sizes and production of O_2_^−^. However, these beneficial effects were reversed by the NADPH oxidase agonist agent TBCA, indicating that the downregulation of NADPH oxidase was involved in the anti-oxidative effect of acupuncture against cerebral ischaemia. Our data are consistent with previous studies that confirmed the role of NADPH oxidase in ischaemic stroke and mild cognitive impairment^22^,^23^,^24^. A recent study reported that electroacupuncture pretreatment attenuated acute cerebral ischaemic injury by inhibiting NAPDH oxidase-mediated oxidative damage in diabetic mice^25^. These findings suggested that NADPH oxidase downregulation by acupuncture attenuated ischaemic oxidative damage in stroke rats, which may represent a novel mechanism of acupuncture-induced neuroprotection against cerebral ischaemia.

It is well established that the overproduction of superoxide anion is a key injurious mechanism during neurodegeneration damage, especially in the context of cerebral ischaemia^9^. Super oxidants have a very short half-life, so it is very difficult to monitor them in real time directly *in vivo*. The most used detection method is DHE staining, which could detect the level of O_2_^−^, the main source of reactive oxygen species. With the minimum values at 6 h, O_2_^−^ was significantly elevated at 96 h as compared to the sham control in acute ischaemic injury^26^. Moreover, significant NADPH activation occurs between 48 and 72 h after a diffuse brain injury^27^ and remains active even at 28 days after a focal brain injury^28^. In the present study, we focused on 14-day acupuncture treatment after cerebral ischaemia. We showed that both NADPH oxidase and its derived O_2_^−^ are significantly enhanced in the 2VO group compared to the normal group, and such an increase was significantly abolished by acupuncture treatment for 14 days after cerebral ischaemia.

RETRACTED

Previous studies provided evidence that gp91phox plays a critical role in ischaemic cerebral damage, and genetic deletion of gp91phox confers protection against ischaemic stroke in mice^29^,^30^. Interestingly, the results in the present research showed that when gp91phox was knocked out, mice showed more impairment in spatial memory after cerebral ischaemia. Furthermore, acupuncture treatment failed to improve memory impairment in gp91phox KO mice. This is in agreement with the study that found that gp91phox subunit knockout mice show a mild deficit in spatial memory under chronic cerebral hypoperfusion^31^. Moreover, it has been demonstrated that NADPH oxidase is expressed in neurons^32^ and localized at synapses^33^. This indicated that NADPH oxidase may be a source of superoxide that is required for normal brain function. Cognitive dysfunction occurs in chronic granulomatous disease patients, which is caused by inherited mutations in genes encoding subunits of the NADPH oxidase complex^34^, suggesting that the lack of a fully functional NADPH oxidase impairs higher-order brain function. We showed that acupuncture could not protect against spatial memory deficits following genetic ablation of gp91phox. Together, these results indicate that acupuncture does require full function of the NADPH oxidase enzyme to protect against spatial memory deficits.

Although multiple investigators have already reported that NADPH oxidase controls oxidative stress in experimental ischaemia, ‘classic’ inhibitor therapy would seem to be of limited usefulness in the treatment of cerebrovascular disease^35^,^36^. One explanation is that successful treatment for preventing the production of O_2_^−^ may require inhibiting multiple isoforms or full NADPH oxidase activity. In addition, the NADPH oxidase inhibitor is likely to be problematic therapy due to lack of selectivity, which could result in the compromise of immune function^37^. Acupuncture inhibits multiple isoforms (gp91phox and p47phox), which provides therapeutic advantages over conventional inhibitors in the treatment of cognitive impairment after ischaemic damage.

Several studies have characterized NADPH oxidase as activated with the translocation/interaction of its cytosolic proteins to the membrane subunit and that it subsequently participates in various pathophysiological mechanisms^38^. In our future research, changes in the levels of NADPH oxidase subunits will be quantified in both the cytosol and the cell membrane fractions extracted from the hippocampus.

RETRACTED

In conclusion, our work provides evidence that acupuncture protects against cerebral ischaemia in two-vessel occlusion rats. These beneficial effects of acupuncture were associated with the attenuation of NAPDH oxidase-mediated oxidative stress. Furthermore, acupuncture requires full function of the NADPH oxidase enzyme to improve cognitive impairment. Our work highlights acupuncture as a potentially promising therapeutic therapy for treatment of cognitive dysfunction in patients with ischaemic diseases. Further clinical trials investigating the effect of acupuncture on cardiovascular outcomes are required to refine our proposal.

## Additional Information

**How to cite this article**: Shi, G.-X. *et al.* Acupuncture elicits neuroprotective effect by inhibiting NAPDH oxidase-mediated reactive oxygen species production in cerebral ischaemia. *Sci. Rep.* **5**, 17981; doi: 10.1038/srep17981 (2015).

## Figures and Tables

**Figure 1:** Acupuncture ameliorated cerebral ischaemia-induced cognitive impairment. Quantification of **(a)** Time latency, **(b)** Swimming distance, **(c)** Swimming speed for reaching the hidden platform during 3 days in hidden platform trial, and **(d)** The percentage of time spent in the target quadrant in probe trial was measured in WKY + Sham, 2VO, 2VO + Acu and 2VO + Non-acu Rats using water maze task. Values are expressed as means ± SEM (n = 10 for each group). *p < *0.05*.

**Figure 2:** Acupuncture suppressed NADPH oxidase-derived ROS generation and attenuated cerebral ischemic injury. Infarct sizes in WKY + Sham, 2VO, 2VO + Acu and 2VO + Non-acu groups. (**a,b**) Photograph of a typical brain slice TTC staining at day 14 after acupuncture treatment and statistical analysis of lesion sizes. Red area is live tissue; white area is dead or dying tissue. (**c**) The ROS generation was determined by DHE staining at day 14 after acupuncture treatment in WKY, WKY + Sham, 2VO, 2VO + Acu and 2VO + Non-acu groups. (**d**) Graphic presentation shows the the NADPH oxidase activity among WKY, WKY + Sham, 2VO, 2VO + Acu and 2VO + Non-acu groups. (**e,f**) Representative images and quantitative graph for Nissl staining in hippocampus’ CA1 region. Values are means ± SEM (n = 10 for each group). *p < *0.05*, **p < *0.01*, ***p < *0.001*.

**Figure 3:** Acupuncture regulated part of NADPH oxidase subunits expression. The expression of different NADPH oxidase subunits at day 14 after acupuncture treatment in WKY, WKY + Sham, 2VO, 2VO + Acu and 2VO + Non-acu groups. (**a–c**) The protein level of p47phox, p67phox, gp91phox and its corresponding GAPDH or β-actin bands were determined using Western blot analysis. The following histogram shows the quantitative densitometry of the blots in each group (n = 6 for each group). **(d)** Graphic presentation shows the expression of gp91phox mRNA level at day 14 after acupuncture treatment analyzed by quantitative RT-PCR (n = 6 for each group).Values are means ± SEM .*p < *0.05*, **p < *0.01*.

RETRACTED

**Figure 4:** The NADPH antagonist mimicked the antioxidant potential of acupuncture, and the NADPH oxidase agonist reversed the beneficial effect of acupuncture. Quantification of (**a**) Time latency, (**b**) Swimming speed and (**c**) The percentage of time spent in the target quadrant in probe trial was measured in 2VO + Acu, 2VO + Vehicle, 2VO + Vehicle + Acu, 2VO + TBCA + Acu and 2VO + Apocynin groups using water maze task. **(d and e)** TTC staining was performed at day 14 after acupuncture treatment. Photograph of a typical brain slice and statistical analysis of infarct sizes. Red area is live tissue; white area is dead or dying tissue. **(f)** ROS generation detected by DHE staining. Values are means ± SEM (n = 10 for each group). *p < 0.05, **p < 0.01, ***p < 0.001.

**Figure 5:** Acupuncture required the full function of the NADPH oxidase enzyme to protect against cognitive impairment. Quantification of **(a)**Time latency, **(b)** Swimming distance, (**c)** Swimming speed for reaching the hidden platform during 3 days in hidden platform trial, and (**d**) The percentage of time spent in the target quadrant in probe trial was measured in WT + VO, WT + VO + Acu, gp91phox + VO and gp91phox + VO + Acu mice using water maze task (n = 10 for each group).Values are expressed as means ± SEM (n = 10 for each group). *p < *0.05*.

**Table 1:** Acupuncture points and manipulations.

Points	Anotomind positions	Manipulation	Twisting angle (degrees)	Frequency (per minutes)	Time (s)
Zusanli (ST36)	2 mm lateral to the anterior tubercle of the tibia, and 5 mm (rat)/3 mm (mice) below the capitulum fibulae under knee joint	Twirling reinforcing manipulation	<90	>120	30
Baihui (DU20)	Midline of the head, approximately midway on the line connecting the apices of the auricles	Twirling reinforcing manipulation	<90	>120	30
Non-acupoints	On the bilateral hypochondrium, 10 mm above iliac crest	Moderate reinforcing-reducing manipulation	90–180	60–120	45
